The article "Rapid Extensive Recurrence of Triple Negative Breast Cancer: Are Both Therapy and Cancer Biology the Culprit?" was published in 2015. Journal: J Clin Med Res.

# Rapid Extensive Recurrence of Triple Negative Breast Cancer: Are Both Therapy and Cancer Biology the Culprit?

**DOI:** 10.14740/jocmr2365w

**Published:** 2015-12-28

**Authors:** Dinesh Vyas, Kaivalya Deshpande, Lakshmishankar Chaturvedi, Laput Gieric, Karen Ching

**Affiliations:** a 61391 ODE Surgery, Department of Surgery, Texas Tech University Health Sciences Center, 3601 Fourth Street, Lubbock, TX 79430, USA; b Michigan State University, College of Human Medicine, 1200 East Michigan Avenue, Suite 655, East Lansing, MI 48824, USA; c These authors contributed equally to this paper.

**Keywords:** Cancer, Doxorubicin, IL-6, Inflammation, Metastasis

## Abstract

Triple negative breast cancer (TNBC) comprises 17-20% of all breast cancers and is one of the most common breast cancers. The lack of therapy and failure of existing therapy has been a challenge for clinicians. Doxorubicin (DOX) is the first-line therapy, however, it has significant limitations. Rapid extensive recurrence with metastasis in any cancer has been a challenge for surgeons and medical oncologists. The challenge can be due to failure of therapy, drug resistance, or epigenetic changes. Here, we are discussing a stage I breast cancer patient, operated and treated with appropriate chemotherapy with complete response, which recurred in less than 8 months and metastasized to bone, liver and other organs. We are also presenting lab data of the IL-6 secretions on exposure to DOX in one of the most commonly used TNBC cell lines MDA-MB-231. Breast cancer cell line MDA-MB-231 upon exposure to DOX shows an increase in IL-6 levels more than the already elevated IL-6 levels. This might be a reason for early recurrence. We concluded that patients with TNBC might benefit from a standard DOX treatment regimen with an inflammation-blocking agent.

## Introduction

Rapid extensive recurrence with metastasis in any cancer has been a challenge for surgeons and medical oncologists. The challenge can be due to failure of therapy, drug resistance or epigenetic changes. Here, we are discussing a stage I breast cancer patient, operated, and treated with appropriate chemotherapy with complete response, seen to recur in less than 8 months and show bone, liver and multiple organ metastasis.

Drug resistance remains a major challenge in cancer therapy. Two broad categories have been identified that classify cancer resistance based on response to chemotherapy: primary and acquired [1]. While primary resistance precedes initial chemotherapy, acquired resistance involves an accumulation of genetic changes following clinical intervention until tumor cells develop resistance phenotypes. A form of acquired resistance is mediated by the interaction of tumor cells with their microenvironment [1]. In this form, tumor cells circumvent the apoptotic effects of chemotherapy through cell-adhesion-mediated resistance, in which tumor cell integrins adhere to fibroblasts or the extracellular matrix [2], and soluble factor-mediated resistance, which induces the stroma to produce cytokines, chemokines, and growth factors [3-5].

The article "Rapid Extensive Recurrence of Triple Negative Breast Cancer: Are Both Therapy and Cancer Biology the Culprit?" was published in 2015. Journal: J Clin Med Res.

## Case Report

A 44-year-old pre-menopausal female presented in August 2012 with a palpable left breast mass which the patient herself first noted weeks prior to first surgical consult. She had no medical problems, no personal or family history of any malignancy. The right breast was unremarkable, and there were no palpable lymphadenopathy (axillary and supraclavicular). A mammogram showed benign right breast and a large asymmetric density in the left breast corresponding to the palpable mass (Fig. 1). She underwent a left needle-localized lumpectomy and left axillary lymph node (LN) dissection. She had PET-CT and MRI showing localized disease (Fig. 2, 3a, c). Final pathology showed pT1N1 disease - stage IIA. The tumor was scattered subcentimeter foci in the lumpectomy specimen with the largest focus measuring 3 mm. She had only one of nine axillary LN with metastatic CA. She then underwent whole breast radiation including axillary, supraclavicular and internal mammary LN basins and concluded the whole course in June 2013.

**Figure 1:** Mammogram. A core biopsy was done of this mass and it showed poorly differentiated triple negative invasive ductal carcinoma.

**Figure 2:** Breast MRI 2012. Given the large triple negative cancer, a breast MRI and PET-CT scan were performed for staging purposes. The PET-CT showed a 5 cm left breast mass which was FDG-avid, as well as an 8 mm left axillary LN and a 5 - 6 mm left internal mammary node both also FDG-avid. No distant metastasis was evident. The left axillary LN underwent an ultrasound-guided biopsy that proved metastatic from the breast. The breast MRI showed a 7.1 × 3.3 cm enhancing mass at the left breast 10:00 - 11:00 position, and a 2.8 cm axillary LN, both of which are already biopsy-proven malignancies. After workup, the patient’s final clinical stage was cT3 N3 M0 - stage IIIC. A multidisciplinary breast conference was held and the group decided that treatment should include neoadjuvant chemotherapy, surgery, whole breast RT including regional basins, and genetic counseling for BRCA testing. The patient underwent six cycles of TAC (docetaxel, doxorubicin and cyclophosphamide) which she finished in January 2013. BRCA testing revealed no mutation in the BRCA 1 and 2 genes. The post-chemotherapy physical exam showed excellent clinical response with no palpable evidence of disease in the left breast. Breast MRI and PET-CT (February 2013) both also showed complete clinical response (both breast tumor and lymphadenopathy). Brain MRI also showed negative findings.

The article "Rapid Extensive Recurrence of Triple Negative Breast Cancer: Are Both Therapy and Cancer Biology the Culprit?" was published in 2015. Journal: J Clin Med Res.

**Figure 3:** PET-CT. (a) Active left breast mass, left ax LN (September 2012). (b) Extensive distant metastasis (July 2013). (c) Active left breast mass (September 2012).

The patient did well but started experiencing some right shoulder, right hip and low back pains. A PET-CT scan was performed in July 2013 to evaluate these symptoms, and showed extensive distant metastasis to include extensive skeletal (axial and appendicular), bilateral lung, liver, left adrenal gland, and extensive cervical, mediastinal and abdominal lymphadenopathy which were all FDG-avid. Liver biopsy was done to confirm the diagnosis and to re-check hormone status of the metastatic lesion. This biopsy confirmed metastatic carcinoma consistent with a primary breast. The hormone receptors were checked and were confirmed triple negative.

### Doxorubicin (DOX) enhances IL-6 production in triple negative MDA-MB-231 breast cancer cells

Cells were exposed to DOX (2 μM) or vehicle (untreated control) for 24 h and secretion level of IL-6 was measured by ELISA in the cultured medium as per manufacturer’s recommendation (BD Biosciences). We observed a basal high level secretion of IL-6 in MDA-MB-231 cells. Cells exposed to DOX significantly further enhanced the production of IL-6 (P < 0.05, n = 3, Fig. 4). This suggests that although DOX is being used as chemotherapeutic agent to treat the breast cancer patients, it somehow enhances the pro-inflammatory cytokine.

**Figure 4:** IL-6 levels significantly increase on 24 h exposure of doxorubicin in triple negative breast cancer cell MDA-MB-231.

## Discussion

### DOX and its limitations

DOX is widely used as an anti-neoplastic drug for hematologic and solid tumors [6, 7]; however, its propensity to cause cardiotoxicity is a major limiting factor [8]. Long-term use of DOX leads to the development of cardiomyopathy and congestive heart failure [9, 10], although the underlying mechanisms remain unclear.

Several reports show that DOX treatment induces inflammation. Furthermore, these studies demonstrate that DOX induces IL-8 [11, 12], NFκB [13], IL-6, TNF-α [11, 14], MCP-112 and G-CSF [14] (Fig. 5). In breast cancer, anthracycline-based chemotherapy is associated with increased levels of inflammatory markers highly relevant in breast tumors such as VEGF, sP-selectin, and vWF [15]. Janelsins and colleagues also demonstrate that cytokine levels of IL-6, IL-8, and MCP-1 are increased in early-stage breast cancer patients who are receiving DOX-based chemotherapy [16]. There is also growing evidence that the inflammatory cytokine IL-1β may play an important role in DOX-induced inflammation. Zhu and colleagues found that serum levels of IL-1β were induced as a result of DOX treatment in mice compared to untreated counterparts, and pretreatment with an IL-1 receptor antagonist prior to DOX treatment protected the mice from DOX-induced mortality and cardiac damage [17]. Sauter and colleagues demonstrated that DOX-induced increased expression of IL-1β is mediated by the activation of NLRP3 inflammasome critical for sensing endogenous danger and stress signals [14].

The article "Rapid Extensive Recurrence of Triple Negative Breast Cancer: Are Both Therapy and Cancer Biology the Culprit?" was published in 2015. Journal: J Clin Med Res.

**Figure 5:** Flowchart of TNBC and doxorubicin.

Several studies also demonstrate that chemotherapy drug effects on adipose tissue may be mediated by DOX-induced activation of NFκB and inflammatory cytokines [18, 19]. Studies on rodent models demonstrated that DOX increases serum total cholesterol, triglyceride and LDL levels when compared to controls [20-22]. Peroxisome proliferator activated receptor gamma (PPAR-γ), a nuclear receptor that acts as a transcription factor, is prominent in white adipose tissue and plays a crucial role in the clearance of serum triglyceride as well as blood glucose [23-25]. From the existing literature, DOX mediates the down-regulation of PPAR-γ [26, 27], which may cause a reduction in the clearance of circulating free fatty acids [28-30], the recruitment of macrophages [31], and thus the activation of NFκB and pro-inflammatory cytokines [32, 33].

#### DOX and metastasis

Several studies have demonstrated that DOX induces EMT acquisition mediated by production of transforming growth factor beta (TGFβ) as well as tumor cell motility. DOX has been shown to induce circulating TGFβ and lung metastasis in xenograft and transgenic animal models. Bandyopadhyay and colleagues showed that DOX treatment in human MDA-MB-231 and murine breast cancer 4T1 cells significantly increased tumor cell migration and invasion [34]. In this study, the investigators explored whether DOX-induced TGFβ production plays a role in tumor cell migration and invasion, and found that similar to TGFβ treatment, DOX treatment enhanced Smad2 and Smad3 phosphorylation in both MDA-MB-231 and murine 4T1 cells, indicating a significant role in EMT-associated signaling. DOX also induced EMT phenotypic characteristics such as spindle-shaped morphology, increased nuclear translocation of Snail, multi-drug resistance protein (MDR1), and formation of mammospheres in murine breast cancer 4T1 cells.

#### Connection between DOX-induced increase in inflammation and metastasis

Recent studies indicate that inflammatory cytokines and the activation of ERK signaling pathways are inextricably linked with tumor growth, progression, invasion, and chemoresistance [18]. A study by Armstrong and colleagues showed that DOX-induced p53 activation in neuroblastoma cell lines is upstream of MEK/ERK pathway, and p53 is necessary for subsequent MEK/ERK signaling resulting in NFκB activation [35]. Elsea and colleagues showed that DOX treatment in murine macrophages resulted in a significant increase in IL-1β and IL-6 mRNA expression and is mediated by the p38 MAPK pathway, indicating a direct role for p38 MAPK in the induction of inflammatory cytokines by DOX [36]. IL-6 and IL-8 in particular have been implicated to play an important role in those with the worst breast cancer prognoses. A recent study by Poage and colleagues suggested that knockdown of both cytokines reduces tumor growth more in triple receptor negative breast cancer (TNBC) than either IL-6 or IL-8 alone [37]. In line with other recent evidence, the study also demonstrated that IL-6 and IL-8 chiefly function through autocrine signaling and activating the NFκB and JAK/STAT pathways, supporting the evidence that these cytokines promote tumor cell propagation, EMT acquisition, and a metastatic phenotype [38, 39]. Taken together, these findings suggest that inflammatory signals may provoke similar effects at the cellular level in promoting tumor cell proliferation and metastasis in breast cancer, although the exact mechanisms implicating DOX-induced metastasis still need to be elucidated.

The article "Rapid Extensive Recurrence of Triple Negative Breast Cancer: Are Both Therapy and Cancer Biology the Culprit?" was published in 2015. Journal: J Clin Med Res.

### Clinical relevance and future direction

It is known that TNBC has various cellular subtypes and they all have varying, and sometimes inconsistent, responses to the first-line recommended chemotherapy. Our efforts highlight the need to understand the limitation of current clinical guideline of treating TNBC as one group and for the most part offering the same standard therapy. Regarding the foreseeable future, it will be insightful to conduct a clinical trial in which IL-6 levels are collected at various treatment stages from patients. The future data will determine if these patients will benefit from anti-inflammatory therapy alongside their chemotherapy to prevent future recurrences.
